The article "Knowledge and attitude of the communities towards COVID-19 and associated factors among Gondar City residents, northwest Ethiopia: A community based cross-sectional study" was retracted in 2026. Reasons: duplicate publication; overlap with earlier publications; concerns about the authorship; concerns about the article.

# Knowledge and attitude of the communities towards COVID-19 and associated factors among Gondar City residents, northwest Ethiopia: A community based cross-sectional study

**DOI:** 10.1371/journal.pone.0248821

**Published:** 2021-04-16

**Authors:** Asefa Adimasu Taddese, Zelalem Nigussie Azene, Mehari Woldemariam Merid, Atalay Goshu Muluneh, Demiss Mulatu Geberu, Getahun Molla Kassa, Melaku Kindie Yenit, Sewbesew Yitayih Tilahun, Kassahun Alemu Gelaye, Habtamu Sewunet Mekonnen, Abere Woretaw Azagew, Chalachew Adugna Wubneh, Getaneh Mulualem Belay, Nega Tezera Assimamaw, Chilot Desta Agegnehu, Telake Azale, Animut Tagele Tamiru, Bayew Kelkay Rade, Eden Bishaw Taye, Zewudu Andualem, Henok Dagne, Kiros Terefe Gashaye, Gebisa Guyasa Kabito, Tesfaye Hambisa Mekonnen, Sintayehu Daba, Jember Azanaw, Tsegaye Adane, Mekuriaw Alemayehu

**Affiliations:** 1 Department of Epidemiology and Biostatistics, Institute of Public Health, College of Medicine and Health Sciences, University of Gondar, Gondar, Ethiopia; 2 Department of Women’s and Family Health, School of Midwifery, College of Medicine and Health Sciences, University of Gondar, Gondar, Ethiopia; 3 Department of Health Systems and Policy, University of Gondar, Gondar, Ethiopia; 4 Department of Psychiatry, College of Medicine and Health Sciences, University of Gondar, Gondar, Ethiopia; 5 Department of Medical Nursing, School of Nursing, College of Medicine and Health Sciences, University of Gondar, Gondar, Ethiopia; 6 Department of Pediatric and Child Health Nursing, School of Nursing, College of Medicine and Health sciences, University of Gondar, Gondar, Ethiopia; 7 School of Nursing, College of Medicine and Health Sciences and Comprehensive Specialized Hospital, University of Gondar, Gondar, Ethiopia; 8 Department of Health Education and Behavioral Sciences, Institute of Public Health, College of Medicine and Health Sciences, University of Gondar, Gondar, Ethiopia; 9 Department of General Midwifery, School of Midwifery, College of Medicine and Health Sciences, University of Gondar, Gondar, Ethiopia; 10 Department of Clinical Midwifery, School of Midwifery, College of Medicine and Health Sciences, University of Gondar, Gondar, Ethiopia; 11 Department of Environmental and Occupational Health and Safety Institute of Public Health, College of Medicine and Health Sciences, University of Gondar, Gondar, Ethiopia; 12 Department of Gynecology and Obstetrics, College of Medicine and Health Sciences, University of Gondar, Gondar, Ethiopia; Health Services Academy Islamabad Pakistan, PAKISTAN

## Abstract

**Background:**

COVID-19 is the novel coronavirus responsible for the ongoing global outbreak of acute respiratory disease and viral pneumonia. In order to tackle the devastating condition of the virus, countries need to attack the virus with aggressive and targeted tactics. Thus, to strengthen the COVID-19 mitigation measures and to give rapid response, there is an urgent need to understand the public’s knowledge and attitude about of the pandemic at this critical moment.

**Objective:**

This study was aimed to assess the knowledge and attitude of communities about COVID-19 and associated factors among Gondar City residents.

**Methods:**

A community based cross-sectional study was done among 623 respondents in Gondar city from April 20-27/2020. Data were collected using a structured questionnaire adapted from different literatures. The data were entered using Epi data version 3.1 and then exported into STATA version 14 for analysis. Bi-variable and multivariable binary logistic regression were performed. Adjusted odds ratio with 95% CI was used to declare statistically significant variables on the basis of p value less than 0.05 in the multivariable binary logistic regression model.

**Results:**

The overall knowledge and attitude of the community towards COVID19 was 51.85% [95% CI (47.91%-55.78%)] and 53.13% [95% CI (49.20, 57.06%)], respectively. In this study, being married [AOR = 0.60 at 95% CI: (0.42, 0.86)], educational level; primary [AOR = 3.14 at 95% CI: (1.78,5.54)], secondary [AOR = 2.81 at 95% CI: (1.70,4.63)], college and above [AOR = 4.49 at 95% CI: 7.92, 13.98)], and family size [AOR = 1.80, at 95% CI: (1.05, 3.08)] were emerged as statistically significant factors impacting the knowledge of the community about COVID-19. Besides, educational level; primary [AOR = 1.76 at 95% CI: (1.03, 3.01)], secondary [AOR = 1.69 at 95% CI: (1.07, 2.68)], and college & above [AOR = 2.38 at 95% CI: (1.50, 3.79)], and family size; four to six members [AOR = 1.84 at 95% CI (1.27, 2.67)], above seven members [AOR = 1.79 at 95% CI (1.08, 2.96)] were factors identified as significantly attribute for positive attitude of the communities towards COVID-19.

**Conclusion:**

More than half of the respondents had better knowledge and attitude regarding COVID-19. Higher educational level and larger family size were significant factors predominantly affecting the knowledge and attitude of the communities towards COVID-19.

## Introduction

In China, Wuhan city, Hubei Province, a cohort of pneumonia cases of unknown cause was reported on December 31 2019 [1]. A novel coronavirus (2019-nCoV) has been incriminated as the cause for the aforementioned disease that has been continuing infecting more than 209 countries with around 1.5 million confirmed cases and 90 thousand deaths globally [2, 3]. In Ethiopia the first case was confirmed on March 13, 2020 [4]. The clinical feature of COVID-19 varies from mild flu like symptoms to severe pneumonia along with acute respiratory distress syndrome, septic shock and multi-organ failure, which in turn leads to in the risk of death. The pandemic (COVID-19) is claimed to be transmitted predominantly from person to person via inhalation the infected aerosols. Other modes of transmissions for the pandemic have also been implicated such as contact with contaminated fomites, and direct person to the infected individual [5, 6].

The COVID-19 disease is spreading drastically in both developed and developing countries including Ethiopia and results in unprecedented catastrophic death and social crisis [7]. The reasons for the high burden of the pandemic in developing nations may ascribed to the limited resources to combat the disease, the use of mass transport, and low awareness of the communities about the disease. Studies, in China and Ethiopia noted that the proportion of communities’ good knowledge about COVID-19 was 90% and 54%, respectively [8, 9]. In Ethiopia, tremendous endeavors are being invested such as developing supportive and reliable informatics, risk assessment and contact tracing activities, laboratory testing, and disseminating information, education, and communication about the diseases through different outlets. However, the pandemic continues to affect the inhabitants of the country even in a more rapid rate.

Moreover, we cannot do community mass screening via blood test to identify the suspected cases, owing to mass transport; mass gathering in religion ceremony and market areas, get limited hygiene and sanitation services.

Therefore, to provide a rapid response against the pandemic, it is imperative to strengthen the taken prevention and control strategies. This calls up on enhancing the communities’ level of knowledge and attitude about the COVID-19. The main aim of this study was therefore to assess the knowledge and attitude of communities about COVID-19 and its associated factors among Gondar City residents, northwest Ethiopia.

## Methods

### Study area

The study was conducted at Gondar city, Amhara regional state, northwest Ethiopia. The city is located at Central Gondar Zone, Amhara regional state of Ethiopia, and is 748 kilometers far northwest of Addis Ababa, the capital of Ethiopia and, about 180 kilometers from Bahir Dar city, the capital of Amhara regional state. It has an altitude of 12°36′N 37°28′E and longitude of 12.60N 37.467’E with an elevation of 2133 meters above sea level and it embraces 12 administrative areas (sub-cities) which consist of 22 kebeles (the smallest administrative unit in Ethiopia). Gondar city is among one of the ancient and largely populated cities in the country. The city has now one public referral hospital and eight governmental health centers.

### Study design and period

A community-based cross-sectional study was conducted from April 20 to 27, 2020.

### Study participants

The source population of this study was all people of age 18 years and above residing in Gondar city while people aged 18 years and higher living in the selected kebeles of the city were the study population.

### Sample size calculation and sampling procedures

The sample size was determined by using single population proportion formula by considering the following statistical assumptions:

Confidence level (Cl), 95%

Proportion = 50%

Margin of error 5%

Using the following single proportion formula:-

$$n=\frac{\left(Za∕2\right)2\;x\;P(1-P)}{(W)2}$$

Where

n = initial sample size

Z = 1.96, the corresponding Z-score for the 95% CI

P = Proportion = 50%

W = Margin of error = 5% = 0.05

$$n=\frac{\left(1.96\right)2\;x\;0.5(1-0.5)}{(0.05)2}=384$$

By considering 10% non-response rate and design effect of 1.5, the final sample size was 635. The participants`households were accessed using cluster sampling technique.

Out of 22 Kebeles, 8 Kebeles (Kebele 7, Kebele 8, Kebele 9, Kebele 13, Kebele 16, Kebele 17, Kebele 18, Kebele 20) were selected by using lottery method. Then from each kebele, one to two Ketena/s (the lowest administrative cluster) were selected depending on the numbers of households. The selected Ketena/s were considered as cluster and all households in the selected Ketena/s were included. Either parents in the household was interviewed or one family member aged above 18 years was the respondent in the household whenever the parents were not available at the time of data collection.

### Operational definitions

#### Information exposure

Respondents were asked whether they heard or not about the various aspects of COVID-19. The responses were coded as yes or no and those who responded median and above score of the information exposure assessment questions were regarded as having good level of information exposure about COVID-19.

#### Good knowledge

Participants who responded median and above score of the knowledge assessment items about COVID-19 were labeled as having good knowledge otherwise poor knowledge about COVID-19.

#### Favorable attitude

Participants who responded median and above score of the attitude questions about the COVID-19 were considered as having favorable attitude towards COVID-19 otherwise unfavorable attitude.

### Study variables

The dependent variables were knowledge and attitude of the communities towards COVID-19. Whereas socio-demographic related variables including sex, age, educational level, family size and communities’ attitude towards COVID-19 preventive measures were the independent variables.

### Data collection tools and procedures

Data regarding the variables were collected through face-to-face interview using a structured questionnaire adapted from different literatures. The respondents were asked about the sources of information about COVID-19 and how much they trust those sources. They were also asked about the types of information that they wanted to receive. Participants were interviewed whether they performed precautionary measures including avoiding handshaking, adopting hand washing, and practicing physical distancing. The full survey questionnaire is provided in the S1 Appendix.

Data were collected by BSc nurses and strictly followed by supervisors who managed the overall data collection process. A one-day training was given to the data collectors and supervisors about the purpose of the study, data collection tools, collection techniques and ethical issues during selection of the study participants and collection of the data. All responses to closed and open questions were written down manually by the interviewers. The supervisors assessed the consistency and completeness of data on a daily basis.

### Statistical analysis

The data entry was performed using the statistical software Epi data version 3.1 and then exported to STATA version 14 for analysis. Descriptive statistics was carried out and presented with narration and tabulation. Binary logistic regression (Bi-variable and multivariable) analysis was performed to identify statistically significant variables using a cut-off p-value < 0.2 in the bi-variable analysis to identify candidate variables for multivariable binary logistic regression. Adjusted odds ratio with 95% confidence interval was used to declare statistically significant variables on the basis of p-value <0.05 in the multivariable binary logistic regression model. Hosmer and Lemeshow goodness of fit test was employed and decision was made at P-value>0.05.

### Ethics approval and consent to participate

Ethical clearance was obtained from the Institutional Review Board (IRB) of the University of Gondar and an official permission letter was gained from the city administrative office. Written informed consent was obtained from each participant before conducting the actual data collection process. Any identifiable issues were eliminated to ascertain confidentiality. Furthermore, appropriate infection prevention practices and principles related to COVID-19 were considered during data collection period. Data collectors provided health education for the household after the interview has been completed based on the gaps identified as appropriate.

## Results

### Socio-demographic characteristics of the study participants

In the current study, a total 623 study participants were involved making the response rate of 98.1%. The median age of the study participants was 33 ± 13.24 (SD) years. Four hundred two (64.53%) of the study participants were females. Three- fifth (59.87%) of the study participants were married. Regarding to the family size of the respondents, t344 (55.22%) had 4 to 6 family members in household. Of the respondents, 202 (32.42%) had attained college and above and 125 (20.06%) had no formal education (Table 1).

**Table 1:** Socio-demographic characteristics of the study participants in Gondar city, northwest Ethiopia, 2020.

Variables		Frequency(n = 623)	Percent (%)
**Sex**	Male	221	35.47
	Female	402	64.53
**Religion**	Orthodox	433	69.50
	Muslim	154	24.72
	Others*	36	5.78
**Age in years**	18 to 26	163	26.16
	27 to 33	150	24.08
	34 to 45	174	27.93
	Above 45	136	21.83
	Median age 33 ± 13.24 (SD)		
**Family size**	Up to 3	178	28.57
	4 to 6	344	55.22
	7 and above	101	16.21
**Educational level**	No formal education	125	20.06
	Primary	101	16.21
	Secondary	195	31.30
	College and above	202	32.42
**Current marital status**	Unmarried	250	40.13
	Married	373	59.87
**Occupation status**	Unemployed	448	71.91
	Employed	175	28.09

*_ Protestant, Catholic, Jewish.

### Prevalence of knowledge about COVID-19

In this study, the overall knowledge of the study participants about COVID-19 was 51.85% at 95% CI (47.91%, 55.78%) (Table 2).

**Table 2:** Knowledge of the study participants about COVID-19 in Gondar city, northwest Ethiopia, 2020.

Variables		Frequency (n = 623)	Percent (%)
**Knowledge about COVID-19 symptoms**	Poor	245	39.33
	Good	378	60.67
**Knowledge about COVID-19 Vulnerability**	Poor	256	41.09
	Good	367	58.91
**Knowledge about COVID-19 prevention measures**	Poor	270	43.34
	Good	353	56.66
**Knowledge about COVID-19 transmission and incubation period**	Poor	256	41.09
	Good	367	58.91
**Overall knowledge**	Poor	300	48.15
	Good	323	51.85

### Prevalence of attitude towards COVID-19

In the current study, the overall prevalence of the communities’ attitude towards COVID-19 was 53.13% at 95% CI (49.20, 57.06%) **(Table 3)**

**Table 3:** Attitude of the study participants towards COVID-19 in Gondar city, northwest, Ethiopia, 2020.

Variables		Frequency (n = 623)	Percent (%)
**Attitude towards COVID-19**	Negative	393	63.08
	Positive	230	36.92
**Attitude towards COVID-19 prevention measures**	Negative	298	47.83
	Positive	325	52.17
**Overall Attitude towards COVID-19**	Negative	292	46.87
	Positive	331	53.13

### Factors associated with knowledge about COVID-19

In our study, those participants who were 40% less likely to have good knowledge about COVID-19 compared to unmarried participants [AOR = 0.60 at 95% CI: (0.42, 0.86)]. Respondents who had attained college and above were 7.92 times more knowledgeable than those who had no formal education [AOR = 7.92, at CI: (4.49, 13.98)]. Respondents who had seven and above family members were 1.80 times more likely to have good knowledge about COVID-19 compared those respondents who had less than three family members [AOR = 1.80, at CI: (1.05, 3.08)] (Table 4).

**Table 4:** Factors associated with knowledge of communities about COVID-19 in Gondar city, northwest Ethiopia, 2020.

Variables		Knowledge		COR at 95% CI	AOR at 95% CI
		Poor	Good		
**Marital status**	Unmarried	103	147	1	1
	Married	197	176	0.63(0.45, 0.87)	0.60(0.42, 0.86)*
**Educational level**	No formal education	93	32	1	1
	primary	50	51	2.96(1.69, 5.19)	3.14(1.78, 5.54)*
	Secondary	100	95	2.76(1.69, 4.50)	2.81(1.70, 4.63)*
	College & above	57	145	7.39(4.46, 12.25)	7.92(4.49, 13.98)*
**Occupational status**	Unemployed	235	213	1	1
	Employed	65	110	1.87(1.30, 2.67)	0.96(0.62, 1.50)
**Family size**	Up to 3	94	84	1	1
	4 to 6	161	183	1.27(0.89, 1.83)	1.47(0.99, 2.16)
	7 and above	45	56	1.39(0.85, 2.27)	1.80(1.05, 3.08)*

AOR = adjusted odd ratio, COR = crude odd ratio, * significant level, * significant at p-value <0.05.

### Factors associated with attitude towards COVID-19

In the multivariable analysis; level of education and family size continued to significantly affect the communities’ attitude towards COVID-19.

In this study, an increased in the level of education has been positively associated with communities’ attitude towards COVID-19 compared to those who had no formal education [primary education AOR = 1.76 at 95% CI: (1.03, 3.01), secondary AOR = 1.69 at 95% CI: (1.07, 2.68), and college & above AOR = 2.38 at 95% CI: (1.50, 3.79)]. Moreover, study participants who had seven and above family members were 1.79 times more likely to have positive attitude towards COVID-19 compared to those who had three and less family members (Table 5).

**Table 5:** Factors associated with attitude of communities towards COVID-19 in Gondar city, northwest Ethiopia, 2020.

Variables		Attitude towards COVID-19		COR at 95% CI	AOR at 95% CI
		Negative	Positive		
**Educational level**	No formal education	74	51	1	1
	Primary	46	55	1.73(1.02, 2.95)	1.76(1.03, 3.01)*
	Secondary	93	102	1.59(1.01, 2.50)	1.69(1.07, 2.68)*
	College & above	79	123	2.26(1.43, 3.56)	2.38(1.50, 3.79)*
**Family size**	Up to 3	101	77	1	1
	4 to 6	146	198	1.78(1.23, 2.56)	1.84(1.27, 2.67)*
	7 and above	45	56	1.63(0.99, 2.67)	1.79(1.08, 2.96)*

AOR = adjusted odd ratio, COR = crude odd ratio, * significant level, * significant at p-value <0.05.

## Discussion

In the current study, we have tried to assess the prevalence of knowledge and attitude of the community to wards COVID-19 and the factors associated with it in Gondar city, northwest Ethiopia. Accordingly, our results yielded that the prevalence of communities’ who had good r knowledge and positive attitude towards COVID-19 were 51.85% at 95% CI (47.91%, 55.78%) and 53.13% at 95% CI (49.20%, 57.06%), respectively.

The prevalence of the study participants with good knowledge is in agreement with earlier reports from Bangladesh [10] and Iran [11] but higher than a study conducted in Ethiopia [12]. The finding of our study (51.85% at 95% CI (47.91%, 55.78%)) however was lower than former evidences reported from Malaysia [13], Vietnam [14], Pakistan [15], Iran [16], Italy [17], Uganda [18], Nigeria [19], Tanzania [20], Pakistan [21], and two studies in China [22, 23]. Regarding to the second outcome of our study, attitude of the communities’ towards COVID-19 (53.13% at 95% CI (49.20%, 57.06%), was lower compared to the findings from Bangladesh [10], Pakistan [20], china [22] and Tanzania [20].

The possible explanations, for the observed discrepancies in the prevalence of knowledge and attitude of the communities’ towards COVID-19 might be ascribed to differences in the study population, tools used to measure the outcome variables across the studies, timing of the study period, the sample size used, the level of information exchange.

In regard to the factors affecting the outcome variables, the socio-demographic variables like marital status, level of education and family size had significantly influenced the knowledge and attitude of the communities’ towards COVID-19. As such, Forty-percent of the respondents who were married were less likely to have good knowledge regarding COVID-19 [AOR = 0.60 at 95% CI: (0.42, 0.86)]. This result is supported by a previous report from China [9]. This could be explained in that those married individuals may carry higher responsibilities to care for their children and their family at large and hence they might be eager to sought for information about the disease thereby they had good knowledge about COVID-19.

Moreover, respondents who attended higher level of education were more likely to have good knowledge and positive attitude compared to those respondents with no formal education [9, 10, 12]. This might be due to the fact that educational attainment is often used as a proxy measure of socio-economic status. And people with higher educational level have better income and have resources to secure information related to the COVID-19 thereby might have good knowledge and positive attitude towards the pandemic. This finding is indicative for policy makers and intervention strategies to focus on community members who have no formal education.

Finally, family size was one of the factors significantly associated with both good knowledge and positive attitude. Cognizant of this, study participants with higher family size were more likely to have good knowledge and positive attitude in the current study. The possible reason for this could be, family members might have discussion about COVID-19 and share information on how to care about each other from the pandemic and this will in turn enable for them to have good knowledge and positive attitude.

### Limitations of the study

This study acknowledged some important possible limitations that should be considered when interpreting the results. First, the study was cross-sectional, a design that does not permit to establish cause-effect relationships. Second, social desirability bias due to self-report might have been introduced.

## Conclusion and recommendation

In the our study, more than half of the study participants had good knowledge and positive attitude towards COVID-19. The socio-demographic variables, such as marital status, level of education and family size were factors significantly affecting the knowledge and attitude of the communities” towards the diseases (COVID-19). We authors recommended that the intervention strategies to halt the pandemic could better provide a due attention on these segments of population including those who had no formal education, unmarried once, households with lower family members.

## Supporting information

S1 Appendix Full survey questionnaire. (DOCX)

S1 Dataset This is the data set used in analysis for the current study. (XLS)

## Abbreviations

AOR: Adjusted Odds Ratio
CI: Confidence Interval
COR: Crude Odds Ratio
COVID-19: Corona virus disease 19
OR: Odds Ratio
SD: Standard Deviation
SPSS: Statistical Package for Social Sciences
TV: Television
WHO: World Health Organization
